This article has been retracted.

# Are Nepali students at risk of HIV? A cross-sectional study of condom use at first sexual intercourse among college students in Kathmandu

**DOI:** 10.1186/1758-2652-13-7

**Published:** 2010-03-02

**Authors:** Ramesh Adhikari

**Affiliations:** 1 Geography and Population Department, Mahendra Ratna Campus, Tribhuvan University, Kathmandu, Nepal; 2 Institute for Population and Social Research, Mahidol University, Salaya, Thailand

## Abstract

**Background:**

Condoms offer the best protection against unintended pregnancies and sexually transmitted infections. Little research has been conducted to determine the prevalence and investigate the influencing factors of condom use at first sexual intercourse among college students.

**Methods:**

A self-administered questionnaire was completed by 1137 college students (573 male and 564 female) in the Kathmandu Valley. Analyses were confined to 428 students who reported that they have ever had sexual intercourse. The association between condom use at first sexual intercourse and the explanatory variables was assessed in bivariate analysis using Chi-square tests. The associations were further explored using multivariate logistic analysis in order to identify the significant predictors after controlling for other variables.

**Results:**

Among the sexually active students, less than half (48%) had used condoms during first sexual intercourse. The results from the logistic regression analysis revealed that age, caste and/or ethnicity, age at first sexual intercourse, types of first sex partner, alcohol consumption and mass media exposure are significant predictors for condom use at first sexual intercourse among the college students. Students in the older age groups who had first sex were about four times (16 to 19 years old) (OR = 3.5) more likely and nine times (20 or older) (OR = 8.9) more likely than the students who had sex before 16 years of age to use condoms at first sexual intercourse.

Moreover, those students who had first sex with commercial sex worker were five times (OR = 4.9) more likely than those who had first sex with their spouse to use condoms at first sex. Furthermore, students who had higher exposure to both print and electronic media were about twice (OR = 1.75) as likely as those who had lower media exposure to use condoms. On the other hand, students who frequently consumed alcohol were 54% (OR = 0.46) less likely to use condoms at first sexual intercourse than those who never or rarely consumed alcohol.

**Conclusions:**

The rate of condom use at first sexual intercourse is low among the students. It indicates students are exposed to health hazards through their sexual behaviour. If low use of condom at first sex continues, vulnerable sexual networks will grow among them that allow quicker spreading of sexually transmitted diseases and HIV. Findings from this study point to areas that policy and programmes can address to provide youth with access to the kinds of information and services they need to achieve healthy sexual and reproductive lives.

## Background

The Federal Democratic Republic of Nepal is a landlocked country in south Asia. It lies between the two of the most populous countries of the world: China in the north and India in the south, east and west. These countries are ranked as the first and the second largest countries of the world, respectively, in size of population. The total population of Nepal was 27.5 million in 2009 [1]. About one in five of Nepal's people are in the age group of 15 to 24 years [2].

HIV/AIDS has become a global problem and has spread all over the world. The latest statistics estimate that approximately 33.4 million people worldwide were living with HIV/AIDS by the end of 2008. Of these, 4.7 million people were in Asia. India, Nepal's neighbour, accounts for roughly half of Asia's HIV prevalence. With the exception of Thailand, every country in Asia has an adult HIV prevalence of less than 1%. However, owing to the region's large population, Asia's comparatively low HIV prevalence translates into a substantial portion of the global HIV burden in terms of numbers [3].

Like other countries in Asia, Nepal is susceptible to HIV. The country is indeed facing critical challenges posed by the rapid spread of HIV/AIDS. By October 2009, about 15,000 cases of HIV infection and about 2600 cases of AIDS had been officially reported. Among these HIV cases, more than two in five cases (41%) were in the college/university-going (15-29 years) age group [4]. However, given the limitations of Nepal's public health surveillance system, the actual number of infections is thought to be much higher. The Joint United Nations Programme on HIV/AIDS (UNAIDS) estimated that 75,000 people were living with HIV at the end of 2007 [5]. It has been found that one in every 200 young males (0.5%) and one in every 300 females (0.3%) aged 15 to 24 are infected by HIV in Nepal [1].

Studies show that college students engage in a variety of behaviours that put them at risk for serious health problems [6,7]. College students are at risk of sexually transmitted infections, including HIV, due to their propensity to take risks, often with multiple partners, accompanied by an inconsistent use of condoms [8,9]. Ample research has also examined the prevalence of excessive alcohol and other substance use, risky sexual behaviour, and other harmful health behaviours that are not uncommon among college students [10-13].

Similarly, a study found that young adults represent one of the groups at highest risk for HIV infection [14]. A study conducted in colleges in Nepal showed that about two in five male college students (39%) had premarital sexual experiences. Among these, more than half reported that they had multiple sex partners. Furthermore, more than one in five (23%) had sexual experience with commercial sex workers, and less than half of them (49%) had used condoms in every act of sexual intercourse with a sex worker [15]. Such risky sexual behaviour increases the risk of contracting an STI or HIV which jeopardizes academic achievement and performance of the students [13,16,17].

Differences in levels of condom use in various population groups and settings have been identified in the literature. In particular, groups with the lowest levels of education have consistently been the least likely to use condoms, both with non-marital and marital partners [18-22]. Some studies also revealed an increase in condom use in the younger age groups [18,23,24] compared to the older groups. Some studies found that later sexual activity has also been associated with an increased use of condoms [25-27]. Furthermore, alcohol use is highly prevalent among college students, and contributes to rising rates of sexual risk taking [28-31]. Empirical evidence also suggests that the mass media has an important role in shaping individual reproductive attitudes and behaviours [32-34]. In fact, the mass media variable is a reliable predictor of condom use among individuals [35,36]. One study showed that men who heard about AIDS through either electronic or print media were 30% to 50% more likely to have used a condom than men not exposed to these media [37].

Many researchers and public health policy makers are particularly interested in the subject of first sexual contact. A person's first sexual intercourse often occurs before the age of 20. This is linked to two factors: the association between behaviours in the first sexual relationship and the establishment of behavioural patterns throughout life [38-40]; and the recognition that sexual initiation at a very young age is a risk factor for pregnancies before the age of 20 and acquiring sexually transmitted diseases, including HIV [26,41].

Condom use at first sex is easily remembered. Some studies have found a strong link between first condom use and lifetime use: a 20-fold increase in lifetime use and a 10-fold increase in current use if a condom was used at first sexual contact [42]. There is a limited body of literature that points to condom use at first sexual contact among young people, especially students, and none of the studies has analyzed the data on condom use at first sex in Nepal.

It is useful to know about condom use during first sexual intercourse in Nepal so that priorities and approaches for interventions to prevent risky sexual behaviour can be better designed. This article aims to determine the prevalence of and investigate the factors associated with condom use at first sexual intercourse among college students in Nepal.

Specifically, it is assumed that students who have sex at an earlier age, who consume alcohol frequently, who have sex with irregular partners, and who have lower exposure to mass media use condoms less at first sexual intercourse. The findings of this study address the gap in knowledge by providing the information on condom use at first sexual intercourse that could assist programme managers of government agencies and non-governmental organizations and the Government of Nepal in designing appropriate and timely education-based interventions in institutions of secondary and higher education.

## Methods

### Data and sampling framework

The data used in this paper comes from a cross-sectional survey on attitude and behaviour towards premarital sex among college students of Kathmandu, the capital of Nepal, carried out in 2006. The survey involved a total of 1137 students (573 male and 564 female) studying in 12 colleges affiliated to Tribhuvan University in Kathmandu. Analyses were confined to 428 students who reported that they have ever had sexual intercourse. The scientific committee, which included the Ethical Review Board of the University Grant Commission in Nepal, approved the proposal and provided funding for this study.

A two-stage random sampling technique was applied. The first stage included a random selection of 12 colleges in Kathmandu. In order to select these colleges, a list of all the private and public colleges affiliated with Tribhuvan University and located in the Kathmandu Valley (which includes three districts: Bhaktapur, Lalitpur and Kathmandu) was obtained from the office of the Vice Chancellor in Kathmandu. This list included colleges that provide intermediate (commonly known as Grades 11 and 12), undergraduate and graduate degrees. In the second stage, two classes were randomly selected from each sampled college. The number of students in a class ranged from 40 to 60. All the colleges are co-educational, and all male and female students present on the day of the interview in the sampled classes were requested to participate in the study.

### Research instrument and data collection

Due to the sensitive nature of the study and the educational background of the respondents, a self-administrated, structured questionnaire in the Nepali language was used to obtain information. The questionnaires were first developed in English and then translated into Nepali. Almost all sections pertaining to the behavioural aspect were based on Behavioral Surveillance Survey questionnaire developed by Family Health International/Impact [43]. However, necessary modifications were made to suit the sample population. The questionnaires were pre-tested among students in a college that had not been selected as part of the study, and later refined as required. The pre-test was conducted to determine whether the questionnaires were in sequential order and the wording in Nepali was understandable or not. Most of the questions were close ended; a few open-ended questions were also included.

Female and male students filled in the questionnaire separately in different classrooms. Each student was allocated a separate bench, as in an exam setting, before the questionnaire was distributed to them. A male researcher supervised the male students' class while a female researcher supervised the female students' class. Students were then requested to place the filled-in questionnaire on a table in the corner of each class.

### Ethical considerations

Before starting the study in a sampled college, approval from the campus administrative authority was obtained. All the participants involved in the study were fully informed about the nature of the study, the research objectives, and the confidentiality of the data. After this, verbal consent was obtained from the participants before they were enrolled in the study. The consent form was also written in the local language, stating the study's objectives, nature of the participant's involvement, risk and benefits, and confidentiality of the data. Students were requested to read the consent form carefully. They were given clear options on voluntary participation. It was also made clear that they could refuse to answer any of the questions and terminate the interview if and when they desired.

All of the approached students agreed to participate in the study. Confidentiality of information was ensured by removing personal identifiers from the completed questionnaires. The names of sampled colleges were not made public and thus, it is not possible for anyone outside the research team to trace reported incidents of sexual behaviour to respondents. Respondents were thus protected from any possible adverse repercussions of participating in the study.

### Variables

The measurable outcome of the study is condom use at first sexual intercourse, a dichotomous variable indicating whether or not the respondent had used a condom during the first sexual encounter.

The independent variables used in the study were: sex of the respondent; age; caste and/or ethnicity; level of education; age at first sexual intercourse; marital status; types of first sexual partner; permanent place of residence; alcohol consumption; mass media exposure; and living arrangement. All these variables were organized into two or three categories, based on those used in other literature, as well as on the frequency distribution of the variables.

The indicators of exposure to mass media include an exposure to radio, television and newspapers. The majority of the students rent rooms in the Kathmandu Valley so it is assumed that not all of them have TVs in their rooms. Thus, radio and TV were combined and treated as electronic media, and newspaper as print media. Almost all students were exposed to at least one type of media (either electronic or print). Because of this, the mass media variable was organized into two categories. If a student was exposed to only one type of media, it was considered as low exposure; if a student was exposed to both print and electronic media, it was considered as high exposure.

Similarly, some ethnic groups in Nepal offer alcohol to the gods in religious ceremonies, and people have to consume alcohol in these ceremonies. Therefore, this variable was categorized into two: (1) never/rarely consume alcohol and (2) frequently consume alcohol (two or three times a week).

The variable, "living arrangement", is also organized into two categories: those students who live with their family members were considered as "with biological family"; those who live away from family members were considered as "without biological family". The other independent variables were categorized in the same way.

### Methods of analysis

All completed survey questionnaires were entered into a database after manual coding and validation. Data entry and validity checks were performed for all the questionnaires by using the computer software programme, dBase IV. The cleaned and validated data was transferred into the SPSS software programme for further processing and analysis.

Both bivariate and multivariate techniques were applied in the analysis. The Chi-square test was used to test the association between the variables. Those variables that were significant in the bivariate analysis were further reexamined in the multivariate analysis (binary logistic regression) in order to identify the significant predictors after controlling for other variables. Before the multivariate analysis, multicollinearity among variables was assessed, and the least important variable, which was highly correlated to other variables, was removed from the logistic model.

## Results

### Characteristics of the respondents

Among the students, about two in five (39%) (47% boys; 28% girls) had sexual intercourse irrespective of their marital status. Among these sexually active students (n = 428), around 27% were aged 15 to 19. Eleven percent reported that they had had sex before the age of 16. A large majority of the sexually active students were from outside of the Kathmandu Valley. More than a third (34%) of the students consumed alcohol frequently (two or three times a week). Almost half of the students resided with their biological families. Almost all students were exposed to at least one type of mass media (either electronic or print). Furthermore, both male and female college students were generally aware of HIV/AIDS and knew of at least one mode of transmission of HIV/AIDS (data not shown).

### Socio-demographics correlate with condom use

Among the sexually active students, just less than half (48%) had used condoms during their first sexual contacts. Table 1 shows the clear association between condom use at first sexual intercourse and different socio-demographic characteristics. Of those who used condoms at their first sex, a significantly higher proportion than their comparison group: were males; were aged 15 to 19; were from the Brahmin and Chhetri communities; had first sex at age 16 or older; were unmarried; had sex with a boyfriend/girlfriend; were from outside the Kathmandu Valley; had high exposure to the mass media; and lived with their biological families (Table 1).

**Table 1:** Condom use at first sexual intercourse by background characteristics (n = 428)

	Condom use			
			
	Yes	No	Percent	Number
Sex of the respondents*				
Female	40.3	59.7	100.0	159
Male	52.0	48.0	100.0	269

Age group**				
15-19	58.6	41.4	100.0	116
20 and above	43.6	56.4	100.0	312

Caste/ethnicity**				
Brahmin/Chhetri	53.1	46.9	100.0	243
Other	40.5	59.5	100.0	185

**Level of education**				
Intermediate	52.3	47.7	100.0	88
Undergraduate	47.2	52.8	100.0	233
Graduate degree	44.9	55.1	100.0	107

Age at first sexual intercourse**				
Up to 15 years	23.4	76.6	100.0	47
16-19 years	50.3	49.7	100.0	195
20 or more years	51.1	48.9	100.0	186

Marital status***				
Married	34.5	65.5	100.0	165
Unmarried	55.9	44.1	100.0	263

Types of first sex partner***				
Spouse	28.9	71.1	100.0	121
Boyfriend/girlfriend	57.2	42.8	100.0	180
Commercial sex worker	52.0	48.0	100.0	127

Permanent place of residence*				
Outside Kathmandu Valley	49.5	50.5	100.0	378
Kathmandu Valley	34.0	66.0	100.0	50

Alcohol consumption*				
Never/rarely consumed	52.7	47.3	100.0	283
Frequently consumed	37.9	62.1	100.0	145

Mass media exposure*				
Low exposure	44.5	55.5	100.0	290
High exposure (both print and electronic media)	54.3	45.7	100.0	138

**Living arrangement**				
With biological family	50.9	49.1	100.0	224
Without biological family (friends/alone)	44.1	55.9	100.0	204

**Total**	**47.7**	**52.3**	**100.0**	**428**

Note: *** = p < 0.001 ** = p < 0.01 * = p < 0.5

Binary logistic regression analysis was used to measure the strength of the association between various independent variables and the probabilities of using condoms at first sex. Only those variables that had significant association in bivariate analysis were reassessed in the logistic model. Before the multivariate analysis, multicollinearity among the variables was assessed. It was found that the variables, "marital status" and "types of first sex partner", were highly correlated (r = 0.7). Therefore, the variable, "marital status", was not included in the logistic model.

Analysis from logistic regression showed that age group, caste and/or ethnicity, age at first sexual intercourse, types of first sex partner, alcohol consumption, and mass media exposure were significant predictors for condom use at first sexual intercourse. Students aged 20 or older were less likely to use condoms (OR = 0.40) than students aged 15 to 19. Similarly, students from castes other than Brahmin and Chhetri were 40% (OR = 0.60) less likely to use condoms during their first sexual intercourses than those from other castes and ethnic groups. Furthermore, students who had sexual intercourse for the first time in the age groups of 16 to 19 and 20 or older were almost four times (OR = 3.5) and nine times (OR = 8.9) more likely, respectively, than students who had first sex before 16 years to use condoms at first sexual intercourse (Table 2).

**Table 2:** Adjusted odds ratio (OR) and 95% confidence interval (CI) for using condoms at first sexual intercourse by selected predictors

Selected predictors	OR	95% CI
**Sex of the respondents**		
Female (ref.)	1.00	
Male	1.34	0.81-2.21

**Age group**		
15-19 (ref.)	1.00	
20 and above	0.40**	0.23-0.71

**Caste/ethnicity**		
Brahmin/Chhetri (ref.)	1.00	
Other	0.60*	0.39-0.94

**Age at first sexual intercourse**		
Up to 15 years (ref.)	1.00	
16-19 years	3.53**	1.58-7.90
20 or more years	8.96***	3.75-21.42

**Types of first sex partner**		
Spouse (ref.)	1.00	
Boyfriend/Girlfriend	4.52***	2.48-8.22
Commercial sex worker	4.98***	2.54-9.74

**Permanent place of residence**		
Outside Kathmandu valley (ref.)	1.00	
Kathmandu valley	0.64	0.32-1.30

Alcohol consumption*		
Never/rarely consumed (ref.)	1.00	
Frequently consumed	0.46**	0.28-0.75

**Mass media exposure**		
Low exposure (ref.)	1.00	
High exposure (both print and electronic media)	1.75*	1.08-2.83

**2 Log likelihood**	**504.68**	

**Cox & Snell R Square**	**0.185**	

Note: *** = p < 0.001 ** = p < 0.01 * = p < 0.5

Those students who had first sex with a commercial sex worker were about five times more likely than those who had first sex with their spouse to use condoms during first sexual intercourse. An inverse relationship was observed between alcohol consumption and condom use. Those students who had frequently consumed alcohol were 54% (OR = 0.46) less likely to use condoms at first sexual intercourse than those who did not consume alcohol. On the other hand, students who had higher exposure to both print and electronic media were about twice (OR = 1.75) as likely as who had lower media exposure to use condoms during their first sexual intercourses (Table 2).

## Discussion

This study shows that condom use at first sexual intercourse is low among college students in Kathmandu, Nepal. If condom use at first sex remains low, vulnerable sexual networks will grow among the students, allowing faster spreading of sexually transmitted diseases and HIV. Our study found that condom use at first sexual intercourse varied according to different criteria. Age group, caste and/or ethnicity, age at first sexual intercourse, types of first sex partner, alcohol consumption and mass media exposure were significant predictors for using condoms at first sexual intercourse.

The study also found that students aged 15 to 19 were more likely to use condoms during first sexual intercourse compared with students aged 20 or older. Results from this study are consistent with those of many other studies [18,23,24]. The finding of this study was also consistent with that of other literature: that later sexual intercourse has also been associated with increased use of condoms [25-27].

Many other studies have found significant differences in condom use according to the type of relationship with sex partners, defined as casual or fixed/steady [44-46]. Our study also supported the finding of other studies that the level of condom use is higher in those who had first sex with casual or non-steady partners than in those who had first sex with spouses or steady partners. Regarding alcohol consumption, results from this study are similar to most other studies: alcohol use contributes to a lower use of condoms and elevated rates of sexual risk [28-31].

Mass media exposure is another important predictor for condom use at first sexual intercourse. Those students who were exposed to both electronic and print media were more likely to use condoms than those who had low exposure to these media. This finding is similar to that of other studies [35,36]. Diffusion theorists postulate that the mass media effect contraceptive use by stimulating partners to discuss contraceptive use [47]. Through the sharing of information and mutual feedback, people give meaning to information, understand each other's views and influence each other [48]. Thus, discussion of contraceptive use leads to the development of a better understanding between partners of their reproductive health goals.

There are some limitations to this study. First, because of the cross-sectional design of the study and the nature of the items used in the logistic regression analysis, the analysis can only provide evidence of statistical association between those items and condom use at first sex and can not show cause-effect relationships. Second, all measures were self-reported. Thus, responses may have been biased by recall errors or intentional misreporting of behaviour. However, the privacy conditions around the study and the use of self-administered questionnaires are likely to have minimized purposeful misreporting.

## Conclusions

The rate of condom use at first sexual intercourse is low among the students. It indicates students are exposed to health hazards through their sexual behaviour. If low use of condoms at first sex continues, vulnerable sexual networks will increase among the students, allowing more growth in the spread of sexually transmitted diseases and HIV.

Our study showed a positive effect of the mass media on condom use at first sex; information about condom use and sexual risk behaviour, including unsafe sex, should be provided through the mass media. Similarly, students who had sex at a later age were more likely to use condoms at first sex. Therefore, awareness programmes that encourage postponement of sexual debuts could benefit the students. Findings from this study point to areas that policy and programmes can address to provide youth with access to the kinds of information and services they need to achieve healthy sexual and reproductive lives.

## Competing interests

The author declares that they have no competing interests.

## Authors' contributions

RA conceived the study and its design, undertook the analysis, and wrote the manuscript.
